# The Impact of Calories Information Displayed on Menus on Fast Food Consumption Among Teachers in Riyadh, Saudi Arabia

**DOI:** 10.7759/cureus.72876

**Published:** 2024-11-02

**Authors:** Manal Abdulaziz Binobead, Naseebah Abdullah Alnafisa, Ghedeir M Alshammari, Naif Mohammed Alotaibi, Sahar Abdulaziz AlSedairy

**Affiliations:** 1 Food Sciences and Nutrition, College of Food and Agriculture Science, King Saud University, Riyadh, SAU; 2 Food Sciences and Nutrition, College of Food and Agriculture Sciences, King Saud University, Riyadh, SAU

**Keywords:** calorie labelling, dietary habits, eating behavior, nutrition awareness, public health

## Abstract

Background

The Saudi population's dietary habits and nutritional patterns have shifted significantly due to rapid industrialization, technological advances, and cultural changes. Fast food, high in calories, saturated fats, and sodium, has become prevalent, contributing to rising rates of obesity and associated metabolic diseases such as type 2 diabetes. To combat this, the Saudi Food and Drug Authority (SFDA) introduced a mandatory menu calorie labeling policy in 2018 to improve public awareness and promote healthier eating choices. However, the impact of this policy on dietary behavior remains mixed and poorly understood.

Methods

This descriptive-analytical study involved 316 male and female teachers in the Riyadh region, selected using stratified random sampling from public and private schools. The study utilized a questionnaire to assess participants' knowledge, attitudes, and practices regarding menu calorie labeling and barriers to its usage. The data were statistically analyzed to explore the association between awareness of calorie labeling and demographic variables.

Results

Most participants (n = 288 (91.2%)) had sufficient knowledge about calorie content in macronutrients, and 234 (74%) found menu calorie information easy to understand. However, misconceptions persisted, with 159 (50.3%) participants unaware that vitamins and minerals do not contain calories. While 175 (55.4%) participants believed that calorie labeling met daily energy requirements, it had a limited impact on weight management or medical condition-related food choices. Females were twice as likely as males to be aware of calorie information (OR: 2.32, *p* = 0.026). Participants who visited restaurants less frequently were more conscious of menu calorie information (*p* = 0.009).

Conclusion

While the SFDA’s calorie labeling policy has increased public awareness, its influence on actual dietary choices remains inconsistent. Many individuals, particularly female teachers, demonstrate awareness of calorie content but do not always incorporate this information into healthier eating practices. The study highlights the need for further educational initiatives to improve understanding and utilization of calorie labeling, especially for individuals with health conditions.

## Introduction

The Saudi population's eating habits and nutritional patterns have significantly changed due to the country's rapid transformation, technological advancements, and cultural instability [1]. Due to society's fast-paced and industrialized nature, the Saudi community has embraced eating out at restaurants, markets, and cafés, resulting in a significant portion of their income, approximately 7.5%, being spent on food and drink services [2].

Among Saudi females, there has been a gradual but consistent increase in the prevalence of overweight or obesity, with rates reaching approximately 65.4% in the eastern region and 70.5% in the western province [3]. In terms of obesity, Saudi men had a lower mortality rate of 43.35% compared to the national average [4]. The incidence of type 2 diabetes mellitus, a severe health condition that is closely associated with obesity, is rapidly increasing in Saudi Arabia, which equates to more than three million people in the population [5].

The changes in the prevalence of overweight, obesity, and related metabolic disorders have been attributed to various social, economic, and lifestyle factors that accompanied the overall increase in per capita income and the recent industrialization of Middle Eastern oil nations. While many interrelated factors contribute to obesity, the imbalance between energy consumed and energy expended is often identified as the main culprit [6]. In addition to inadequate calorie intake, other factors contributing to being overweight include practices that disrupt metabolism and the consumption of less nutrient-dense foods that promote fat storage [7].

Calorie display through menu labeling is a widely recommended strategy to reduce global obesity and related chronic diseases, whereas, in many countries, governmental policies have primarily focused on highlighting the calorie content of food [8]. In developed countries such as the United Kingdom, as part of the government's Responsibility Deal, food retailers are required to provide consumers with calorie information [9]. In Brazil, major fast-food chains have started listing calorie information on their menus, and municipalities and states are working to pass legislation mandating menu labeling [10].

Despite these initiatives, consumers may still seek information on calorie content without fully understanding what the term "calorie" means. Even those who claim to understand calories may not consistently make the best choices when dining out at restaurants [11]. However, the results of studies on the impact of providing calorie counts in restaurants on customers' food choices have been mixed. While some studies have shown that customers choose healthier options with fewer calories when this information is available, they may also perceive the healthiest options to be the ones with the lowest calorie counts. Conversely, some studies have found limited evidence to support the hypothesis that providing customers with calorie counts in a restaurant reduces calorie consumption or increases healthier dining options overall [12,13]. However, there has been a recent recommendation that the focus of menu labeling policies should shift from solely reducing obesity rates to promoting healthy eating habits overall [14]. This is because nutritional health involves a complex interplay between dietary habits, nutrients, and other nutritional components [15].

In Saudi Arabia, the Saudi Food and Drug Authority (SFDA) introduced a regulation on menu calorie labeling in August 2018 [16]. By December 2018, the SFDA mandated that cafeterias, dine-in restaurants, fast-food outlets, establishments selling fresh squeezed juices and pastries, educational institutions, and government agencies prominently display calorie information on their menus. Several studies evaluated public awareness, attitudes, perceptions, and behaviors regarding this mandatory menu calorie labeling policy. However, the findings were mixed, showing varied impacts on consumer dietary habits [14]. Therefore, this research aimed to evaluate teachers' level of awareness, barriers, and practice towards calorie information on menus, as well as understanding and general interest in consuming meals away from home. It also examined the relationship between the level of awareness and consciousness towards health and demographic characteristics.

## Materials and methods

Study design and population

This descriptive-analytical study involved a sample of 316 male and female instructors from various schools in the Riyadh region. The sample included randomly selected instructors from kindergarten, primary, intermediate, secondary, and special education levels, spanning both public and private institutions within Riyadh and its affiliated governorates.

Data collection 

Data were collected from teachers who completed their education during the second semester of the year 1440/1441 AH. Stratified random sampling was used to select participants. A structured questionnaire served as the data collection tool, consisting of two main sections. (i) Demographic variables: age, gender, educational level, and income. (ii) Cognitive axes: assessment of teachers' interest in calorie information displayed on food menus, knowledge, attitudes, practices, and barriers.

The questionnaire included 45 questions, grouped into categories such as awareness versus non-awareness and consciousness versus non-consciousness regarding calorie information on menus. To culturally adapt the instrument, the questionnaire was translated into Arabic using a forward-backwards translation method. A pilot study was conducted to validate the tool, which achieved a reliability score of 0.856.

Data processing and statistical analysis

The collected data were entered into an MS Excel file (Microsoft® Corp., Redmond, WA) and then exported into SPSS 25.0 (IBM Corp., Armonk, NY) for analysis. The data were categorized into two groups: aware versus not aware and conscious versus non-conscious of calorie information. Descriptive statistics such as the mean, median, standard deviation, and range were used to summarize the quantitative data. Chi-square tests were applied to analyze relationships between variables, and frequency and percentage measures were used throughout the analysis. Logistic regression was employed to determine the association between the level of awareness and demographic characteristics, with a significance level set at p<0.05.

## Results

Participant demographics

This study included 316 participants, with the majority being women (n = 275, 87%) and men accounting for 13% (n = 41). The age distribution of the participants revealed that 124 (39.2%) were aged between 31 and 40 years, 119 (37.7%) were aged between 41 and 50 years, 43 (13.6%) were aged between 20 and 30 years, and 30 (9.5%) were aged between 51 and 60 years. Regarding educational background, 101 (32%) had completed primary school, 87 (27.5%) had completed intermediate school, 86 (27.2%) had completed high school, 27 (8.5%) had attended kindergarten, and 15 (4.7%) had received special education. Regarding household income, 134 (42.4%) participants reported earning between 10,000 and 15,000 SAR monthly. Additionally, nearly half of the participants were categorized as overweight or obese, with 120 (38%) and 109 (34.5%) of participants falling into these categories based on their BMI readings (Table 1).

**Table 1:** Demographic characteristics of the participants. Data were expressed as numbers (N) and percentages (%).

Variables		Frequency (N=316)
Gender	Male	41 (13%)
	Female	275 (87%)
Age (years)	20–30	43 (13.6%)
	31–40	124 (39.2%)
	41–50	119 (37.7%)
	51–60	30 (9.5%)
Social status	Single	27 (8.5%)
	Married	264 (83.5%)
	Divorced	14 (4.4%)
	Widowed	11 (3.5%)
Educational level	Kindergarten	27 (8.5%)
	Primary stage	101 (32%)
	Intermediate stage	87 (27.5%)
	High school	86 (27.2%)
	Special education	15 (4.7%)
Monthly income (in SAR)	<5000	58 (18.4%)
	5000–10,000	76 (24.1%)
	10,000–15,000	134 (42.4%)
	15,000–20,000	48 (15.2%)
BMI level (kg/m^2^)	Underweight (<18.5 kg/m^2^)	4 (1.3%)
	Normal weight (18.5–24.9 kg/m^2^)	83 (26.3%)
	Overweight (25–29.9 kg/m^2^)	120 (38%)
	Obesity (≥30 kg/m^2^)	109 (34.5%)

Knowledge of menu calorie labeling

The results regarding participants' knowledge about calorie labeling on menus are shown in Table 2. Most participants demonstrated sufficient knowledge of menu calorie labeling, particularly in understanding calories. Two hundred and eighty-eight (91.2%) participants knew that carbohydrates, proteins, and fats contain calories, while 234 (74%) participants reported that the calorie information on restaurant menus was easy to understand. However, some areas of knowledge deficiency were identified. One hundred and fifty-nine (50.3%) participants were unaware that vitamins and minerals do not contain calories, while 144 (45.6%) believed incorrectly that 1 g of fat contains the same calories as 1 g of sugar.

**Table 2:** Assessment of knowledge towards menu calorie labeling. Data were expressed as numbers (N) and percentages (%).

Knowledge of menu calorie labeling		Aware	Not aware
1	Calories measure the amount of energy in food.	265 (83.8%)	13 (4.1%)
2	Calculating the calories consumed in food helps to reach a healthy weight.	277 (87.6%)	12 (3.8%)
3	Vitamins and minerals contain calories.	58 (18.3%)	159 (50.3%)
4	Carbohydrates, proteins, and fats contain calories.	288 (91.2%)	7 (2.2%)
5	One gram of fat contains the same number of calories as one gram of sugar.	66 (20.9%)	144 (45.6%)
6	An individual's calorie needs are determined based on several factors: weight, height, age, gender, and physical activity.	279 (88.3%)	3 (0.9%)
7	The Food and Drug Authority obligated restaurants and cafes to display calorie information on the list of foods.	282 (89.2%)	1 (0.3%)
8	It is recommended to look at the calorie information when ordering food from a restaurant.	280 (88.6%)	2 (0.6%)
9	Calorie information displayed on restaurants' menus is easy to understand.	234 (74%)	18 (5.7%)
10	Adults need an average of 2,000 calories per day.	176 (55.7%)	17 (5.4%)
11	Individual calorie needs vary from person to person.	285 (90.2%)	3 (0.9%)
12	Knowing the calorie count helps to balance the added energy and the energy used in the body.	274 (86.7%)	3 (0.9%)

Attitudes toward menu calorie labeling

Table 3 highlights participants' attitudes toward menu calorie labeling. One hundred and seventy-five (55.4%) participants agreed that calorie labeling on menus helped meet daily energy requirements. However, displaying calorie information on menus was not perceived to contribute to weight gain or loss. Participants with medical conditions did not significantly rely on calorie information to make informed food choices.

**Table 3:** Assessment of attitudes towards menu calorie labeling. Data were expressed as numbers (N) and percentages (%).

Attitudes toward calorie labeling		Yes	No	Maybe	I don't know
1	Writing calories on menus helps in weight management.	82 (25.9%)	142 (44.9%)	75 (23.7%)	17 (5.4%)
2	Writing calories on menus meets daily energy requirements.	175 (55.4%)	30 (9.5%)	81 (25.6%)	30 (9.5%)
3	Use calorie information because of a medical condition.	82 (25.9%)	234 (74.1%)	0 (0%)	0 (0%)

Practices regarding menu calorie labeling

Table 4 illustrates participants' behaviors toward calorie labeling. Most participants demonstrated a good level of consciousness about menu calorie labeling. Two hundred and seventy-nine (88.3%) reported that eating healthy food was important. Two hundred and seventy-two (86%) agreed that consuming fruits and vegetables twice a day was important. Two hundred and thirty-five (74.3%) emphasized the importance of low-fat meals. However, the study also found that 150 (47.5%) participants did not care if the snacks they consumed were healthy, 149 (47.2%) did not consistently follow a healthy and balanced diet, and 134 (42.4%) ate food without worrying whether it was healthy, and they did not avoid meals high in cholesterol.

**Table 4:** Assessment of practices towards menu calorie labeling. Data were expressed as numbers (N) and percentages (%).

Practices toward calorie labeling		Conscious	Not conscious
1	I do not care about healthy food when eating.	129 (40.8%)	125 (39.6%)
2	I care a lot about eating healthy food.	219 (69.3%)	23 (7.3%)
3	I eat the food I like without bothering if the food is healthy or not.	134 (42.4%)	112 (35.5%)
4	It is important that the meals I eat are low in fat.	235 (74.3%)	24 (7.6%)
5	I always eat a healthy, well-balanced diet.	149 (47.2%)	64 (20.3%)
6	It is important that my meal is high in vitamins and minerals.	219 (69.3%)	19 (6%)
7	I do not care if the snacks are healthy or not.	150 (47.5%)	86 (27.2%)
8	I do not avoid meals if they are high in cholesterol levels.	116 (36.7%)	124 (39.2%)
9	I believe that knowing how to eat nutritious foods is critical.	279 (88.3%)	7 (2.2%)
10	I think other people care more about healthy meals than I do.	183 (57.9%)	40 (12.6%)
11	I think it is important to eat fruits and vegetables twice a day.	272 (86%)	14 (4.4%)
12	I care about not eating too much food.	221 (69.9%)	24 (7.6%)
13	I care a lot about eating a balanced diet.	230 (72.8%)	13 (4.1%)
14	I care a lot about eating my meals regularly.	205 (64.8%)	24 (7.5%)
15	I avoid eating an amount of sugar.	215 (68%)	34 (10.8%)

Ninety-seven (30%) participants reported that the calorie information on menus was not written. When asked if they spent a lot of time reading calorie information when choosing meals, 56 (17.7%) said "Yes," and 25% said "Maybe" (Table 5).

**Table 5:** Barriers towards menu calorie labeling. Data were expressed as numbers (N) and percentages (%).

Barriers towards menu calorie labeling		Yes	No	Maybe	I don't know
1	Calories in menus are usually written clearly.	97 (30.7%)	97 (30.7%)	95 (30.1%)	27 (8.5%)
2	Spend a lot of time reading calories when choosing a meal.	56 (17.7%)	169 (53.5%)	79 (25%)	12 (3.8%)

Demographic influence on awareness and consciousness

The practices of participants about their demographic characteristics revealed that females were more aware and conscious of menu calorie labeling than males (p < 0.044). Individuals who visited restaurants less frequently (less than once per week) were more conscious of menu calorie labeling (p = 0.009). However, this association decreased as the frequency of restaurant visits increased (p = 0.003), even after the mandatory menu calorie display was implemented.

Logistic regression analysis

The logistic regression analysis found that Females were twice as likely to be aware of menu calorie labeling compared to males, with an odds ratio of 2.32 (CI: 1.10-4.87, p =0.026). No significant association was found between other demographic characteristics and awareness or consciousness of menu calorie labeling (Table 6).

**Table 6:** Association between participants' knowledge and practices with demographic characteristics. Data were expressed as numbers (N) and percentages (%). ^#^One-way ANOVA. *Significant at P <0.05.

Variables		N	Knowledge			Practice		
			Aware	Not aware	*P*-value#	Conscious	Unconscious	*P*-value#
Gender	Male	41	36 (87.8%)	5 (12.2%)	0.37	17 (41.5%)	24 (58.8%)	0.044*
	Female	275	253 (92%)	22 (8%)		160 (58.2%)	115 (41.8%)	
Age (years)	20–30	43	39 (90.7%)	4 (9.3%)	0.689	23 (57.3%)	20 (46.5%)	0.177
	31–40	124	114 (91.9%)	10 (8.1%)		71 (57.3%)	53 (42.7%)	
	41–50	119	107 (89.9%)	12 (10.1%)		61 (51.3%)	58 (48.7%)	
	51–60	30	29 (96.7%)	1 (3.3%)		22 (73.3%)	8 (26.7%)	
Social status	Single	27	25 (92.6%)	2 (7.4%)	0.37	14 (51.9%)	13 (7.4%)	0.499
	Married	264	243 (92%)	21 (8%)		150 (56.8%)	114 (48.1%)	
	Divorced	14	11 (78.6%)	3 (21.4%)		9 (64.3%)	5 (43.2%)	
	Widowed	11	10 (90.9%)	1 (1.9%)		4 (36.4%)	7 (63.6%)	
Educational level	Kindergarten	27	25 (92.6%)	2 (7.4%)	0.969	13 (48.1%)	14 (51.9%)	0.746
	Primary stage	101	93 (92.1%)	8 (7.9%)		53 (52.5%)	48 (47.5%)	
	Intermediate stage	87	78 (89.7%)	9 (10.3%)		52 (59.8%)	35 (40.2%)	
	High school	86	79 (91.9%)	7 (8.1%)		50 (58.1%)	36 (41.9%)	
	Special Education	15	14 (93.3%)	1 (6.7%)		9 (60%)	6 (40%)	
Monthly income (in SAR)	<5000	58	55 (94.8%)	3 (5.2%)	0.496	31 (53.4%)	27 (46.6%)	0.57
	5000–10,000	76	68 (89.5%)	8 (10.5%)		44 (57.9%)	32 (42.1%)	
	10,000–15,000	134	124 (92.5%)	10 (7.5%)		79 (59%)	55 (41%)	
	15,000–20,000	48	42 (87.5%)	6 (12.5%)		23 (47.9%)	25 (52.1%)	
BMI level (kg/m^2^)	Underweight (<18.5 kg/m^2^)	4	4 (100%)	0 (0%)	0.479	2 (50%)	2 (50%)	0.925
	Normal weight (18.5–24.9 kg/m^2^)	83	75 (90.4%)	8 (9.6%)		45 (54.2%)	38 (45.8%)	
	Overweight (25–29.9 kg/m^2^)	120	113 (94.2%)	7 (5.8%)		70 (58.3%)	50 (41.7%)	
	Obesity (≥0 kg/m^2^)	109	97 (89%)	12 (11%)		60 (55%)	49 (45%)	
Frequency of visiting a restaurant during the week before implementing this decision	≤1	194	181 (93.3%)	13 (6.7%)	0.174	118 (60.8%)	76 (39.2%)	0.009*
	2	50	46 (92.0%)	4 (8%)		30 (60%)	20 (40%)	
	≥3	72	62 (86.1%)	10 (13.9%)		29 (40.3%)	43 (59.7%)	
Frequency of visiting a restaurant during the week after implementing this decision	≤1	107	192 (93.3%)	15 (7.2%)	0.104	127 (61.4%)	80 (38.6%)	0.003*
	2	51	48 (94.1%)	3 (5.9%)		29 (56.9%)	22 (43.1%)	
	≥3	58	49 (84.5%)	9 (15.5%)		21 (36.2%)	37 (63.8%)	

## Discussion

While personalized eating habits are crucial for improving health, establishing a favorable national environment is equally important for promoting and expanding healthy eating behaviors [17]. National laws and regulations related to health and the food industry can significantly influence dietary choices at the societal level in Saudi Arabia. Therefore, it is valuable to investigate the impact of the implementation of Strategy 2030 by the Saudi Food and Drug Authority (SFDA), which mandates the display of calorie information on menu options to reduce detrimental eating patterns associated with non-communicable diseases [18]. However, participants in this study do not always practice these habits, often consuming high-calorie snacks without considering their nutritional value and failing to avoid them despite being aware of their high fat and cholesterol content.

Our findings align with a survey conducted by Washi in the UAE, which revealed that many customers (89.5%) are aware of the need to check nutrition labels, yet they are often reluctant to do so; they typically do not utilize calorie information on menus when selecting meal options, focusing instead on basic details like manufacturing and expiry dates [19]. These results suggest that individuals may be concerned about their inadequate knowledge of nutrition, particularly their ability to interpret dietary information for informed nutritional decisions. Despite the SFDA's efforts to enhance nutritional awareness, limited research exists on daily calorie information provided on menu options and other consumption habits among Saudi adults [20]. Our data indicates that only 25.9% of respondents "usually" utilize calorie information from restaurant menus. In contrast, Alkhaldy et al. reported that although Saudi customers strongly support the policy requiring calorie content on menus, these same individuals indicated they would be less likely to dine in restaurants that offered such information [14].

Another notable finding of this study is that teachers spend considerable time reading calorie information when choosing meals [21]. These findings are consistent with studies conducted elsewhere. A previous study found that 51% of respondents surveyed at food stalls utilize calorie information provided on menus to make meal selections, a tendency that may vary based on the menu layout aimed at promoting low-calorie meals [22]. The theory of planned behavior (TPB) suggests that attitudes and shared beliefs predict rational thought regarding choice behavior [23]. Our data indicate a link between mindset and the use of calorie information on menu options, consistent with previous research by Kim et al., which found that attitude impacts customer intention [24].

AlShehri and AlMarzooqi observed that one factor hindering individuals from selecting meals based on calorie information displayed on menus is their inability to comprehend calorie counts, along with their inadequate understanding of how to use calorie information effectively [25]. Additionally, many individuals expressed concern that tracking calories might prevent them from fully enjoying their food. Haynos and Roberto found that although calorie counts influenced most learners when selecting food portions, individuals were also affected by other factors [26]. Affordability was the most critical factor in their selections, followed by meal components and, lastly, meal quantity.

Interestingly, our study findings indicated that females were more aware and health-conscious regarding menu calorie labeling. This aligns with findings from Artica et al., which indicated that females are more inclined to choose healthy food based on published nutritional information [27]. This has been corroborated by other research showing that females are more likely than males to examine calorie labels and nutrition information [28]. Our study contributes to the growing body of research on the impact of menu calorie labeling on consumer food choices [13]. However, despite efforts to provide more nutritious menu options, inconsistencies in the effectiveness of calorie labeling have been noted, revealing gaps in understanding how visual aids influence healthy food choices [29].

## Conclusions

A balanced and appropriate diet is essential for the health of individuals, families, and society, particularly in early childhood, as children learn habits that benefit them throughout their lives. Based on the current study's findings, one of its most important recommendations is to educate teachers on the significance of providing accurate and comprehensive nutrition education to enhance public awareness and understanding of menu calorie labeling. Additionally, this research highlights the lack of association between calorie labeling and weight gain, as well as the limited use of calorie information by individuals with medical conditions, suggesting a need for further education and awareness-raising initiatives. There are several limitations to this explanatory study. First, the study was limited to teachers in Riyadh City, which restricts the generalizability of the findings. Secondly, the study relied on participants' perceptions, knowledge, attitudes, and practices regarding calorie information displayed on menus, which introduces the possibility of inherent subjective bias. Lastly, the study is limited by its small sample size; future research should aim to achieve greater statistical power by utilizing larger sample sizes.

## Figures and Tables

**Figure 1:** IRB approval letter

## Appendices

The effect of calories written in menus on the consumption of fast food for teachers in the city of Riyadh. Dear teachers, none of you is aware of the importance of food in human life, moderation in eating, and not being extravagant. In this sense, instructions were recently issued by the competent authorities to compel restaurants and food stores to write calories on menus and food products. Based on that, we wanted to know the effect of these instructions on fast food consumption on the teachers’ segment in the city of Riyadh. So, I hope you will answer this questionnaire. I pledge to maintain the confidentiality of the information, and it is intended for scientific research purposes only. Researcher: Naseebah Abdullah Abdullwahab Al-Nafisah Email: 438203577@student.ksu.edu.sa.

**Table 7:** Questionnaire.

Questions						
1	Gender	Male	Female			
2	Age (years)	20-30	31-40	41-50	51-60	>60
3	Social status	Single	Married	Divorced	Widowed	
4	Weight (kg)					
5	Height (cm)					
6	The highest educational stage	Kindergarten	Primary	Intermediate	High School	Special Education
7	Do you suffer from any of the following diseases?	Obesity.	Diabetes.	Blood pressure.	Heart disease.	None.
8	Physical activity	I don't do any activity.	Light activity (housework or half an hour walks 3 or less times a week).	Moderate activity (walking an hour or going to the gym 3-4 times a week).	High activity (running or swimming in the club an hour a day 4-5 a week).	
9	Would you like to increase your physical activity in the future?	Yes	No	Maybe		
10	What do you think of the new decision of the competent authorities to compel restaurants and food stores to write calories on their menus?	Awesome, and I loved it.	Good.	Not good.	I don't care.	
11	When ordering from the restaurant, do you specify the type of food because the calories in it are lower than some other foods?	Yes.	No.	Maybe.		
12	Do you think that forcing restaurants to do so will help the community to choose healthy food in the future?	Yes.	No.	Maybe.	I don’t know.	
13	When you visit restaurants, what is the thing that catches your attention the most when reading the menu?	Price.	Description of the meal.	Shape.	Calories.	
14	Are calories in menus usually written clearly?	Yes.	No.	Maybe.	I don’t know.	
15	Do you spend a lot of time reading calories when choosing a meal?	Yes.	No.	Maybe.	I don’t know.	
16	After committing this decision, did you become more attentive when purchasing a meal with the number of calories in it?	Yes.	No.	Maybe.	I don’t know.	
17	How many times do you visit the restaurant during the week before obligating this decision? Please select the time.					
18	How many times do you visit the restaurant during the week after obligating this decision? Please select the time.					
19	Do you think writing calories on menus will help you maintain your weight?	Yes.	No.	Maybe.	I don’t know.	
20	Do you think writing calories on menus will help you lose weight?	Yes.	No.	Maybe.	I don’t know.	
21	Do you think writing calories on menus will help you gain weight?	Yes.	No.	Maybe.	I don’t know.	
22	Do you think that writing calories on menus meets daily energy needs?	Yes.	No.	Maybe.	I don’t know.	
23	Are you using calorie information because of a medical condition?	Yes.	No.			
24	Do you calculate your daily calorie intake?	Yes.	No.			
26	Please indicate how much you agree with the following phrases: (Knowledge)					
	Phrase	Strongly Agree	Agree	Neutral	Disagree	Strongly Disagree
	1- Calories are a measure of the amount of energy in food					
	2- Calculating the calories consumed in food helps to reach the appropriate weight					
	3- Vitamins and minerals contain calories					
	4- Carbohydrates, proteins and fats contain calories					
	5- One gram of fat contains the same number of calories as one gram of sugars					
	6- An individual's calorie needs are determined based on factors including weight, height, age, gender and physical activity.					
	7- The Food and Drug Authority obligated restaurants and cafes to display calorie information on the list of foods					
	8- It is recommended to look at the calorie information when ordering food from the restaurant					
	9- Calorie information displayed in restaurants is easy to understand					
	10- Adults need an average of 2,000 calories per day					
	11- Individual calorie needs vary from person to person					
	12- Knowing the number of calories helps to balance the added energy and the energy used in the body					
27	Please indicate how much you agree with the following phrases: (Practice)					
	Phrase	Strongly Agree	Agree	Neutral	Disagree	Strongly Disagree
	1- I don't care about healthy meals when eating					
	2- I am very concerned that the food I eat is healthy					
	3- I eat the food I like without caring whether the food is healthy or not					
	4- It is important that the meals I eat are low in fat					
	5- I always follow a healthy and balanced diet					
	6- It is important that my meal be high in vitamins and minerals					
	7- I don't care if snacks are healthy or not					
	8- I do not avoid meals if they raise cholesterol levels					
	9- I think it is very important to know how to eat healthy food					
	10. I think other people care more about healthy meals than I do					
	11- I think it is important to eat fruits twice a day and eat vegetables					
	12- I take care not to eat much food					
	13- I am very interested in eating a balanced diet					
	14- I take great care to eat my meals regularly					
	15- I take care to avoid eating an amount of sugar					
